# Research on Modular Management of Railway Bridge Technology Innovation in Complex and Difficult Mountainous Areas

**DOI:** 10.1155/2022/8799586

**Published:** 2022-08-11

**Authors:** Huihua Chen, Qintao Cheng, Yingxue Xie, Chaoxun Cai, Xinlin Ban, Xiaodong Hu

**Affiliations:** ^1^School of Civil Engineering, Central South University, Changsha 410083, Hunan, China; ^2^Guangzhou Municipal Engineering Design & Research Institute Co.,Ltd., Guangzhou 510000, China; ^3^China Academy of Railway Science Corporation Limited, Beijing 100081, China

## Abstract

With China's government facilitating railway projects, more railway bridges (RBs) are gradually built in complex and difficult mountainous areas (CDMAs). The construction activities of RB in CMDAs are facing formidable challenges in terms of the natural environment, technology, and organization management, which are hardly solved by traditional bridge design and construction techniques. Therefore, there is an urgent need for technology innovation (TI). Studies on the management of RB-TI in CMDAs are limited. As such, this study aims to offer an effective modular management approach to RB-TI in CMDAs. A system of demand and obstacle factors for RB-TI in CMDAs was identified firstly based on the literature review and the grounded theory, including seven intermediate codings and 29 initial codings. Then these factors were regarded as the system requirements for modular decomposition, to establish a “cut-to-fit” modular management approach to RB-TI in CMDAs. A case (i.e., the LD bridge project of the CZ railway) was selected to demonstrate and validate the developed approach. The results show that the proposed approach can be applied to manage RB-TI in CMDAs. The innovation of this study lies in the integration of grounded theory and modular theory and provides modular management ideas and measures for bridge engineering technology innovation. Findings from this study enrich the knowledge body of RB-TI and guide innovation subjects in the practical management of RB-TI in CMDAs.

## 1. Introduction

In recent years, China's national railway network has been improved and gradually penetrated CMDAs in the western of the country. Due to the large number of mountains and ravines to be crossed, the form of “railway replacing with bridges” is adopted in many lines. As a result, the bridge project accounts for a high proportion of the railway project in China [1]. By the end of 2019, the number of high-speed railway bridge projects in China exceeded 10,000, with a total length of about 16,000 km, accounting for 45.2% of the entire length of railway lines [2]. It was validated that the form of “railway replacing with bridges” can substantially deal with complex geological conditions, reduce foundation settlement, protect the environment, and improve line flatness [3]. Therefore, the bridge project is of crucial importance for the smooth construction of the railway.

Complex and difficult mountainous areas refer to mountainous areas with harsh natural environments, significant terrain height differences, complex geological conditions, strong tectonic activities, strict environmental protection requirements, weak infrastructure, and relatively difficult construction environments. China's CMDAs are mainly located in the Qinghai-Tibet Plateau, the Yunnan-Guizhou Plateau, and the Sichuan Basin. When building RBs in these areas, they need to face the more complex and difficult natural environments such as complex wind fields of gorges, extreme geological hazards, and harsh climates. They are also characterized by long construction periods, discontinuous construction cycles, complex interests, and high demands for collaboration in terms of organization and management. For instance, the LD Bridge project in the CZ railway is a typical example of them and the complex and difficult mountainous environment makes its construction process full of challenges. However, in the context of the challenges brought by environmental characteristics and bridge characteristics, the traditional RB design and construction technology are hard to overcome so many challenges to satisfy the actual needs, so TI is urgently needed.

With the raising of innovative awareness of the whole society, the concept of TI gradually draws more researchers' attention. According to Liu et al. [4–6], vigorously promoting TI can effectively save costs, improve the competitiveness and economic benefits of enterprises, and achieve sustainable development. For this reason, it is of great importance to promoting TI of RB projects in CMDAs. RB-TI in CMDAs is the deepening and extension of existing bridge engineering design and construction technologies, as well as the development of new technologies that may emerge in the future. According to the literature review, there are abundant achievements in RB-TI, which mainly focus on structural design [7, 8], construction technology [9, 10], maintenance [11, 12], and intelligent construction [13, 14], etc. However, few researchers have studied the management of TI in bridge projects during railway construction, and this has led to the low efficiency of TI. As a result, we need to develop a systematic and comprehensive approach to managing RB-TI in CMDAs.

Although no existing studies specifically focus on the management approach of RB-TI in CMDAs, previous literature can identify many management methods of TI that can provide a methods pool for this study, such as modular theory, TRIZ theory, analytic hierarchy process (AHP), structural equation model (SEM), and work breakdown structure(WBS). For instance, Qi and Wu [15] established an integrated innovation network for low-carbon technologies on modular; Ding et al. [16] proposed a design framework for the construction TI platform based on TRIZ to improve the innovation capacity and efficiency of the industry; Liu [17] applied AHP to develop an analytical model for the TI competitiveness of the regional high-tech industry in China; Jiang et al. [18] employed SEM to analyze the paths of influence of humble leadership on the innovation of technology standards. TRIZ theory can quickly and accurately analyze and identify core problems to improve the efficiency of innovation, but it tends to ignore the role of the innovation subject and its characteristics. Although AHP can determine the main factors affecting innovation efficiency, it lacks effective management tools. Additionally, SEM provides a way to analyze the impact path of technology innovation rather than a management method. In general, all three methods focus on analysis instead of management.

Modular theory is one of the effective strategies for designing and organizing complex products or processes. The theory was proposed by Simon (1962) and developed into a systematic stage of research by Baldwin and Clark et al. [19, 20]. The merit of this method is that it can help simplify complex systems and increase their level of standardization, specification, and refinement. As a result, modular theory has been widely applied to product development [21], TI [22], strategic management [23], and industrial development [24]. At present, modular theory is still in the process of development, and the theoretical system is not yet completed [25]. As such, many researchers have combined modular theory with other methods to increase its practicality. Grounded theory is a qualitative research method. The method was initially proposed by Strauss and Glaser (1987) in response to field observations of doctors dealing with the dying patient, aiming at constructing a theory from empirical data without theoretical assumptions. Since then, the method has been widely exploited as a theoretical research method in many research areas, such as psychology [26, 27], sociology [28, 29], and management [30, 31]. The reason is that grounded theory can derive a substantive theory from empirical data, and then obtain a formal theory from the substantive theory, which can guide theoretical research in a new field without theoretical guidance [32]. Modular theory can be combined with grounded theory, and the multi-level conceptual system constructed by grounded theory can provide the basis for the decomposition and integration of modular theory, thus improving the applicability and relevance of modular management.

Based on the literature review, this paper focuses on the modular management of RB-TI in CMDAs. The objectives of this study are: (1) To analyze and refine the demand and obstacle factors of RB-TI in CMDAs through grounded theory to provide system requirements for modular decomposition. (2) To establish a modular management approach to RB-TI in CMDAs by applying modular theory. (3) To demonstrate and validate the developed method through a case study. The study can enrich the management theory of RB-TI during railway construction in CMDAs by providing a modular management approach. Besides, from the practice point of view, this study can facilitate the management of RB-TI by project developers, designers, constructors, and other stakeholders. The developed method can improve the efficiency of RB-TI in CMDAs and relieve the pressure on the subjects of TI, which will promote the standardized management of RB-TI in CMDAs.

## 2. Methodology

This study mainly applies grounded theory and modular theory to conduct research on the modular management of RB-TI in CDMAs. Firstly, the collected empirical data are coded in layers with grounded theory to refine and analyze the demand and obstacle factors of RB-TI in CDMAs, thereby clarifying the system requirements for modular decomposition. Next, based on the established decomposition principles and system requirements, modular theory is introduced to decompose RB-TI in CDMAs in a modular way, which will provide the basis for the subsequent establishment of modular management ideas and approaches. The detailed workflow of this study is shown in Figure 1.

### 2.1. Grounded Theory

Grounded theory is a qualitative research method developed for social scientific research, that aims to develop a theory grounded in empirical data [33]. The first step of this method is to collect and select the data in the research field. Then, we need to analyze the essence of things and phenomena hidden in the data to refine the core concepts of nature and identify the complex relationships between them. After that, we can construct a relevant theory through the categorization of core concepts with coding layer by layer based on their relationships [34].

Though grounded theory must be supported by empirical evidence, its main characteristic is not in its empirical nature but in the fact that it abstracts new concepts and ideas from empirical facts. It can fully combine literature, field data, or interview records to refine important concepts and obtain effective information. It allows for empirical generalizations to be drawn directly from practical observation without theoretical assumptions in the process of collecting and analyzing information. At last, the generalizations can rise to a theory with universal applicability.

At present, there are only a few studies on RB-TI in CDMAs, and no perfect theory can be used to guide the research. This also leads to the fact that people cannot comprehensively and systematically consider the obstacles to be overcome and the demands to be fulfilled when managing RB-TI in CDMAs, which results in TI being out of touch with reality and inefficient. The first task of this study is for this reason to identify the system requirements for the modular management of TI. By using grounded theory, we can reduce, transform and abstract the huge empirical data into concepts and establish a multi-level conceptual system of the demand and obstacle factors of RB-TI in CDMAs, to promote the research on its modular management of it.

First of all, a large amount of data was collected in this study before applying grounded theory to ensure that the data adequately cover all demand and obstacle factors of RB-TI in CDMAs. Secondly, the collected data were coded layer by layer, especially in three stages: initial coding, intermediate coding, and advanced coding [35].

#### 2.1.1. Initial Coding

Analyze original literature and case materials word by word and sentence by sentence. Then select original phrases or paraphrase them in the researcher's own words to enter the data. Afterward, attempt to discover the initial concept class generic, i.e., initial coding.

#### 2.1.2. Intermediate Coding

Analyze the result of initial coding to discover the relationship between each initial concept class generic, e.g., subordination and causality. According to the relationship, the concept categories can be developed on the basis of the initial coding, i.e., intermediate coding.

#### 2.1.3. Advanced Coding

Analyze every intermediate coding and discover one or more core categories. The core categories are characterized by their ability to encompass most concept categories within a relatively broad theoretical.

Finally, the coding situation needs to be tested for saturation, and those that do not pass the test continue to be coded with additional data until they pass the test, resulting in a final coding situation. The specific operation process is shown in Figure 2.

### 2.2. Modular Theory

The main idea of modular theory is to decompose a complex system into different sub-modules, define the work content of each sub-module, and provide a management way for the modular internal and modules' connection.

There are many types of modular management. Pine II [36] classified modular management into the shared component modular, the interchangeable component modular, the “cut-to-fit” modular, the BUS modular, etc. As the railway bridge project is unique as a construction project, the modular management methods of different RB projects cannot be directly applied and need to be adjusted according to the actual situation. Therefore, this paper adopts the “cut-to-fit” modular, i.e., the modular decomposition and module functions are customized according to the system requirements of the RB project, and the functions of each module are clarified, thus achieving a personalized, targeted, and adaptable modularity. The system requirements are determined by grounded theory in the previous step.

The application of the “cut-to-fit” modular in RB-TI in CDMAs enables each sub-module to show strong professionalism and convenience when running. Furthermore, it can also maximize the engineering efficiency and promote the project tends standardization and institutionalized management based on satisfying the quality requirements of RB engineering in CDMAs.

Hence, we take the demand and obstacle factors system of TI derived from grounded theory as a reference and select the list of demands and obstacles to be exceeded for TI according to the actual situation of different RB projects from it. Exactly, these demands and obstacles form the system requirements for modular management. Based on these system requirements, and combined with certain decomposition principles, we can decompose the complex system of RB-TI in CDMAs into several sub-modules that can work independently. Afterward, the content of each sub-module is specified, and management advice is proposed for the management of the modular internal and modules' connection.

## 3. Case Study

### 3.1. Case Description

The Luding Bridge (LD), located in Luding County, Sichuan Province, is one of two kilometer-long railway suspension bridges spanning deep gorges in the CZ railway. The LD Bridge spans the Dadu River, with the main girder span of 1280 m, a deck elevation of 1680.415 m, and a maximum bridge height of 370 m. It is a suspension bridge with steel truss girders. Besides, the main cable of the LD Bridge adopts prefabricated parallel steel wire strands with a strength class of 1960 MPa, and the main girder is lifted in one section by a cable crane. Additionally, the stiffening beam is a top-bearing steel joist with a main joist center distance of 30 m. The main tower is a reinforced concrete main tower, with a height of 262 m and a height of 141 m. The foundation of the tower is based on a group of large diameter bored piles, and a high-power rotary drilling rig is planned for construction. The anchor is a tunnel anchor with a long guide tunnel and is proposed to be excavated using the drill and blast method. Furthermore, the construction period of the LD Bridge is approximately 66 months. A rendering of the LD Bridge is shown in Figure 3.

### 3.2. Application of Grounded Theory

#### 3.2.1. Data Collection

In this step, we focused on 17 pieces of literature and 10 cases from a large number of data with a high degree of relevance to this study, as shown in Tables 1 and 2.

#### 3.2.2. Initial Coding

Through the initial coding of literature and case data collected above, 29 factors of demand and obstacles of RB-TI in CMDAs are summarized, illustrated in Table 3.

#### 3.2.3. Intermediate Coding

After continuously analyzing the subordination and causality between the 29 initial codings and creating relationships between them, seven intermediate codings are obtained, which are demands of survey and design TI, demands of construction TI, demands of maintenance TI, external environmental obstacles, technology management obstacles, resource use obstacles, and organization management obstacles. The results of the intermediate coding are presented in Table 4.

#### 3.2.4. Advanced Coding

Based on the intermediate coding, further generalization and upgrading are carried out. And finally, two advanced codings with a high degree of generalization and overview are obtained, i.e., demands of TI and obstacles of TI. The detailed coding results are depicted in Figure 4.

#### 3.2.5. Saturation Test

By searching on the web of science, 10 representative pieces of literature on RB-TI in CMDAs were screened for hierarchical recoding. The final result indicated that the result of initial codings did not change, only the expression of some of the codings differed. At the same time, two doctoral students and two master's students in the research team were invited to independently complete the initial coding and test based on the reliability calculation formula proposed by Boyatzis [54]. The calculated reliability is 0.93, which is greater than the basic requirement of 0.70 proposed by Boyatzis. As such, it is considered that the selection of demand and obstacle factors of RB-TI in CMDAs is basically in line with the theoretical saturation test.

#### 3.2.6. Demand and Obstacle Factors of the LD Bridge's TI

The LD Bridge crosses through a steep mountainous area with high mountains, deep valleys, complex geological conditions, and high seismic intensity. At the same time, the bridge has a large span and high piers. Based on these practical characteristics, and combined with the multi-level conceptual system of demand and obstacle factors of RB-TI in CMDAs, we select six demands and five obstacles of TI from the system. The demands include wind-resistant design, seismic design, environmental design, anchor construction, deep water construction, and integration of construction and maintenance. The obstacles consist of challenging construction on steep slopes, difficult lifting of stiffened beam sections, large project size, difficulty in transporting materials, and a high level of risk management. See Table 5 below for a detailed analysis.

### 3.3. Modular Analysis of the LD Bridge TI

#### 3.3.1. Decomposition Principles

Under the guidance of the research objectives, the following principles of modular decomposition are formed by combining the characteristics of RB in CMDAs:

- Keep the sub-modules independent of each other;
- Ensure the realization of module functions;
- Conform to the structural characteristics of suspension bridges;
- Focus on accuracy and scientificity;
- Fit the actual production life.

#### 3.3.2. Modular Decomposition of the LD Bridge TI

According to the above principles and the “cut-to-fit” modular, we decompose the system of the LD Bridge TI into 8 sub-modules based on the demands and obstacles of the project TI, which are as follows: TI module of canyon wind resistance, TI module of strong seismic resistance in the near field area, TI module of environmental protection, TI module of deep water operation, TI module of the construction of large tunnel anchors, TI module of steep slope construction, TI module of stiffened beam section lifting, and TI module of structural durability. Besides, for the three remaining obstacles, i.e., large project scale, difficulty in transporting materials, and high level of risk management, we can adopt modular management measures such as modular decomposition and modular connection management. The details of the modular decomposition of the LD Bridge TI are shown in Table 5.

#### 3.3.3. The LD Bridge TI Module and Its Work Content

According to the system requirements, we divide the LD Bridge TI system into 8 sub-modules. The next step is to clarify the work content of each sub-module so that they can function independently and be integrated according to certain rules to serve the innovation system.

*(1) TI Module of Canyon Wind Resistance.*The LD Bridge is located in a deep “V” shaped canyon mountainous area. Influenced by the topography and atmospheric flow, it is significantly different from the conventional wind field environment, featuring high average wind speed, high turbulence intensity, high wind angle of attack, and high gust coefficient. Therefore, the existing bridge wind design specifications are no longer applicable. At present, the main methods to obtain the wind field characteristics of the deep “V” canyon bridge site area are field measurements, wind tunnel tests, and numerical simulations. Due to the existing technical constraints, it is difficult to accurately simulate the wind field characteristics of the deep “V” canyon by simple wind tunnel tests and theoretical derivation. As a result, the TI module of canyon wind resistance is incorporated into the LD Bridge TI modular system. In this module, we need to undertake on-site wind environment and wind characteristics observation, “wind-vehicle-line bridge” coupling vibration analysis research, to provide technical protection for the LD Bridge against canyon wind performance and train safety operation. In addition, in order to reduce the adverse effects of canyon wind and increase the safety performance of traffic, structural measures and pneumatic measures can be employed.

*(2) TI Module of Strong Seismic Resistance in the Near Field Area.*There are many fracture zones along the CZ railway line, so the bridge structure faces the threat of a near-fault earthquake. Near-fault seismic intensities are large and differ significantly from conventional earthquakes, which makes it difficult to accurately consider the effects of near-fault earthquakes in bridge design. The LD Bridge site is located in a high-intensity seismic zone, with a peak acceleration of 0.30 g and a characteristic period of 0.6 s. The project seismic design takes into account the effect of vertical ground shaking and increases the design of vertical anti-falling beam devices. At the same time, the topography of the LD Bridge is very different in height, with steep slopes and deep valleys, so the topographical effects of ground vibrations at the different piers need to be considered. Combined with the above characteristics, the TI module of strong seismic resistance in the near field area is incorporated into the LD Bridge TI modular system to research on seismic performance and vibration isolation measures for large-span railway suspension bridges in CDMAs.

*(3) TI Module of Environmental Protection.* The ecological environment around the LD Bridge is fragile, so TI related to environmental protection is very important. Therefore, the TI module of environmental protection is incorporated into the LD Bridge TI modular system, realizes the assembly of bridge components, and reduces the impact on the surrounding atmospheric environment, water environment, and ecological environment. In this module, we need to firstly uphold the attitude of respecting nature and establish the idea of harmonious development between humans and nature. According to this, we then should develop new methods of RB construction through TI to minimize the impact on the ecological environment and ensure ecological balance and harmony.

*(4) TI Module of Deep Water Operation.* TI module of deep water operation is the technical innovation of deep water operation platform construction of the LD Bridge project. The LD Bridge crosses the Dadu River, which has a deep water level. During the construction of the abutments of the LD Bridge, the strength, stability, and solidity of the construction platform, which is located in the deep water area, are strictly checked and carefully calculated using innovative technology or means.

*(5) TI Module of the Construction of Large Tunnel Anchors.* The geology of the LD Bridge anchor site area is weakly weathered diorite, broken weakly weathered diorite, and fractured rock interlayer. The use of tunnel anchors in these areas involves a series of technical problems such as the excavation of tunnel chambers, the bearing capacity, and deformation of tunnel anchors, which need to be investigated through thematic studies and scientific research. Hence, the TI module for the construction of large tunnel anchors is incorporated into the LD Bridge TI modular system. In this module, we need to conduct a series of studies, including the study of the LD Bridge tunnel anchor pull-out bearing capacity and force mechanism, the study of the support scheme for tunnel anchor construction, the study of the stability of the surrounding rock, the evaluation of the reinforcement effect, and the verification of the field scale down model test.

*(6) TI Module of Steep Slope Construction.* During the construction of the LD Bridge, the foundation burial depth is large and the soil layer on both banks is hard, so the original foundation construction technology is no longer applicable. So the TI module of steep slope construction is also incorporated into the LD Bridge TI modular system. In this module, because the construction of the foundation and tunnel anchors on both sides of the LD Bridge is a multi-layer crossover operation of different heights, active protection fences, passive protection fences, and profile steel support structures need to be installed to ensure the smooth construction of the LD Bridge project.

*(7) TI Module of Stiffened Beam Section Lifting.* The LD Bridge is located in a high mountainous area with very steep terrain on both sides, extremely inaccessible, and a narrow site, making it impossible to transport stiffened beam sections by water. Therefore, stiffened beam sections could not be lifted from the valley floor and there are difficulties in the actual construction. For this reason, the TI module of stiffened beam section lifting is also incorporated into the LD Bridge TI modular system. The bars are transported individually to the tower position and then lifted. While the mid-span steel girders are first taken from the tower, then lifted symmetrically from the main span toward the tower, and finally, the girders are brought together at the tower root.

*(8) TI Module of Structural Durability.* The LD Bridge is in a location with strong ultraviolet rays, large temperature difference, poor climatic conditions, thin air, difficult to arrive personnel and poor conditions for later operation and maintenance. The LD Bridge is also of great social and political significance, serving as an important channel for multi-ethnic communication and harmony. Consequently, the TI module of structural durability is incorporated into the LD Bridge TI modular system. In this module, we need to take effective measures for the durability of the steel girders, main cable system, anchorage system, and main towers of the LD Bridge to extend their service life. At the same time, attention should be paid to the quality of the LD Bridge and related structural deformation monitoring during operation and maintenance to realize the integration of construction and maintenance.

### 3.4. The Modular Management Measures of the LD Bridge TI

Through modular decomposition and integration, we clarify the work contents, functions, and innovation goals of each sub-module. Below we will put forward the measures of modular management from three aspects to improve the modular management model, i.e., internal management measures for TI module, management measures between TI modules, and management measures for the connection of the TI module with other modules.

#### 3.4.1. Internal Management Measures of TI Module

Based on the long duration, a large number of participating subjects, the extremely complex natural environment, and the high schedule and cost control requirements of the LD Bridge, we propose the following four aspects of internal management measures of TI module: (1) build a multi-body collaborative innovation model; (2) establish a modular parallel engineering coordination model on TI; (3) construct a modular management platform; and (4) follow the principle of experimentation first in TI.

#### 3.4.2. Management Measures between TI Modules

In the construction process of LD Bridge, the determination of module standards is the most critical factor when different TI modules are connected. For example, when the eight TI sub-modules mentioned above are promoting the task of TI, one of the major reason for the frequency of conflicts is the lack of uniformity in the standards of the modules. This also leads to substandard quality of engineering interfaces, thus affecting the overall TI efficiency and engineering quality of RB projects in CMDAs. Consequently, to solve the problems associated with the TI modular management of the LD Bridge from a technical management perspective, unifying the standards of each module is the most crucial measure.

#### 3.4.3. Management Measures for the Connection of the TI Module with Other Modules

The TI module and other modules are mainly managed in three ways: technology management, resource management, and team management. Technology management includes strict design change management, optimization of construction organization design, and unification of technical standards of each module. Resource management consists of planning multiple material transportation routes, promoting standardized material management, ensuring sufficient supply, and reserve of human resources, and supporting risk management through contract groups. Team management includes opening up multiple communication channels, training and induction of modular managers, and improving the assessment, reward, and punishment system.

### 3.5. Results Analysis and Practice Implications

Through grounded theory, we get a total of 29 demand and obstacle factors of RB-TI in CMDAs, which indicates that the traditional management methods are not well adapted to RB projects in CMDAs and not conducive to TI in the projects. Therefore, modular theory can be introduced to study the modular decomposition and modular management of RB in CMDAs oriented towards TI.

Combined with the actual characteristics of the LD Bridge, from 29 demand and obstacle factors of TI, we select six demands of TI, i.e., wind-resistant design, seismic design, environmental design, anchor construction, deep water construction, and integration of construction and maintenance, and five obstacles of TI, i.e., challenging construction on steep slopes, difficult lifting of stiffened beam section, large project size, difficulty in transporting materials, and high level of risk management. These demands and obstacles are the chief problems, we need to address in applying modular theory.

Based on the established decomposition principles and the “cut-to-fit” modular, we divided the system of the LD Bridge TI into eight sub-modules according to its system requirements, including the TI module for canyon wind resistance, TI module for strong seismic resistance in the near field area, TI module of environmental protection, TI module of deep water operation, TI module of the construction of large tunnel anchors, TI module of steep slope construction, TI module of stiffened beam section lifting, and TI module of structural durability. These eight TI modules are functionally independent of each other. By clarifying the work content of each sub-module, we can improve the efficiency of TI, disperse the pressure on innovation subjects and increase the level of standardized management.

Finally, we suggest measures for modular management of RB-TI in CMDAs in terms of three aspects: internal management measures for TI module, management measures between TI modules, and management measures for the connection of the TI module with other modules, to improve the modular management model and provide a reference for practical project applications.

The successful implementation of modular management of TI in the LD Bridge project is a breakthrough in the field of project management, as the application of modular theory in project practice is relatively infrequent. Therefore, according to the current Chinese laws and regulations on project construction, the relevant industry standards, and the various documents in the process of TI in the LD Bridge project, a “guide to the modular management of engineering technology innovation” can be formulated. In addition, the modular connection is one of the more complicated issues, so there are rather particular problems with it in practice. For such problems, a special management team can be set up to formulate special treatment plans and take targeted measures to reduce conflicts and contradictions, which is conducive to the smooth construction of the project and the achievement of management goals. At the same time, study the common practice of modular management, implement modular management in the construction process of more engineering projects, and promote technological innovation.

## 4. Conclusions and Recommendations

This paper proposed a novel approach to modular management for RB-TI in CMDAs. A multi-level conceptual system of demand and obstacle factors of RB-TI in CMDAs was established based on the previous pieces of literature and project cases through grounded theory, which could serve as the basis for system requirements of modular decomposition. The demand and obstacle factors can be integrated into seven categories: survey and design, construction, maintenance, external environment, technology management, resource use, and organization management. Additionally, there are 29 second-ordered demand and obstacle factors of RB-TI in CMDAs under the seven categories. Through modular theory, the decomposition of RB-TI in CMDAs in a modular way is carried out by taking large span suspension bridges as an example, thus establishing modular management of RE-TI in CMDAs based on demands and obstacles, which can effectively promote engineering innovation.

We utilized the LD Bridge to exemplify the practical applicability of the developed approach. The case study indicates that there are mainly eight TI sub-modules in the LD Bridge project, which are the TI module of canyon wind resistance, TI module of strong seismic resistance in the near field area, TI module of environmental protection, TI module of deep water operation, TI module of the construction of large tunnel anchors, TI module of steep slope construction, TI module of stiffened beam section lifting, and TI module of structural durability. By clarifying the content of each module, the developed approach points out the direction for project participants to carry out TI, which will lead to greater efficiency and standardization. In addition, modular management measures are proposed from three aspects: internal management measures for TI module, management measures between TI modules, and management measures for the connection of the TI module with other modules, thus improving the modular management model and providing a reference for practical project applications.

The constructions of this study are as follows: (1) This study enriches the engineering management theory of RB construction, especially on the management of TI; (2) a systematic and comprehensive multi-level conceptual system of demand and obstacle factors of RB-TI in CMDAs is proposed for the first time and this clearly defines the direction of RB-TI in CMDAs; and (3) a modular management approach for RB-TI in CMDAs has been established and the approach can guide project developers, designers, constructor, and researchers to manage the RB-TI in CMDAs, thereby improving the efficiency and standardized management of TI.

However, there are three limitations to this study: (1) There are many types of RB in CMDAs, and this paper only takes large span suspension bridges as an example to explore the ideas and ways of modular management of TI; (2) we only applied the approach into one RB project, and more complete TI modules can be identified in other RB projects; (3) We mainly carried out the qualitative analysis, and future research can evaluate the technological innovation capability of RB projects on this basis, so as to better promote technological innovation management. Thus, we suggest future research can be focused on the abovementioned aspects.

## Figures and Tables

**Figure 1:** The framework of the study.

**Figure 2:** Process of grounded theory.

**Figure 3:** The LD Bridge rendering.

**Figure 4:** Detailed coding on factors influencing RB-TI in CMDAs.

**Table 1:** Literature related to the demands and obstacles of RB-TI in CMDAs.

No.	Author	Main content
1	Wei [37]	Analyze the dilemma faced by the technical management of road bridge construction and propose management strategies.
2	Q. Wang and L. Zhang [38]	Introduce the technical breakthroughs and technical management measures and effectiveness of three major bridge projects in the Yunnan, Guizhou, and Sichuan regions.
3	Wang [39]	Explain the key technical factors affecting the construction of railway bridges and propose relevant quality control measures.
4	Cao [40]	Analyze the elements and countermeasures or the maintenance technology of large span suspension bridges systematically.
5	Lei et al. [41]	Elaborate on the key technologies of high-speed railway bridge construction in China.
6	He et al. [42]	Introduce the main achievements and key technologies of high-speed railway bridges in China in recent decades.
7	Han [43]	Analyze the factors affecting the construction technology of road bridges in terms of people, materials, and machines.
8	Sun [44]	Study the factors affecting the construction technology of road bridges and the corresponding countermeasures.
9	Ci and Tan [45]	Analyze the technical points of the construction of the main cables of complex mountainous railway bridges by taking the beipan river bridge as an example.
10	Li [46]	Analyze the important and difficult points in the construction technology of a super-long span railway suspension bridge.
11	Wu et al. [47]	Describe the design method, calculation theory, and the corresponding technical standards of high-speed railway suspension bridges in China.
12	Su et al. [48]	Review the recent practices of high-speed railway bridges in China and Germany and discuss the development trends.
13	Xiao [49]	Apply AHP to comprehensively assess the technical condition of complex mountain railway bridges.
14	Guo [50]	Study the factors influencing the innovation capability of large and complex engineering technology and the mechanism of enhancing it.
15	Liu et al. [51]	Elaborate on the key technical issues of large span bridges.
16	Jiang [52]	Take the ChaHe bridge as the case base to study the optimization measures for the bridge engineering design of the Shanghai-Kunming railway.
17	Liao et al. [53]	Use the MaAn Moutain bridge as an example to study the design and construction of bridge tower foundations in deep water operations.

**Table 2:** Cases of long-span suspension bridges in CMDAs.

No.	Bridge name	Span (m)	Bridge Height (m)	Category	Mountainous area	Year
1	The baling river bridge	1088	370	Road bridge	Guizhou, China	2009
2	The Sidu river bridge	900	496	Road bridge	Hubei, China	2009
3	The Aizhai bridge	1176	336	Road bridge	Hunan, China	2012
4	The Pulite bridge	628	500	Road bridge	Yunnan, China	2015
5	The Qingshui river bridge	1130	406	Road bridge	Guizhou, China	2016
6	The Dimu river bridge	538	360	Road bridge	Guizhou, China	2016
7	The long river bridge	1196	280	Road bridge	Yunnan, China	2017
8	The Hulukou bridge	656	211	Road bridge	Sichuan, China	2017
9	The Xingkang bridge	1100	285	Road bridge	Sichuan, China	2018
10	The Jinsha river bridge	660	250	Railway bridge	Yunnan, China	2020

**Table 3:** The demand and obstacle factors of RB-TI in CMDAs.

No.	Initial coding	Literature source	Data source
1	Wind-resistant design	10, 16	1–10
2	Seismic design	2, 6, 8	4, 7, 8
3	Environmental design	1, 13, 16	7, 10
4	Anti-fatigue design	13, 16	1–10
5	Main cable erection	3, 6	1–10
6	Strong wind construction	2, 8	1–10
7	Optimization of materials and equipment	7, 9, 10	2, 3, 10
8	Deep water construction	17	5, 7
9	Eco-friendly construction	9, 13	4, 5, 7, 10
10	Anchor construction	8, 10	1–10
11	Monitoring and measuring	8, 14	9, 10
12	Corrosion protection	4, 7, 13	1–10
13	Integration of construction and maintenance	1, 4, 11	10
14	Emergency plans	4, 11, 13	5, 8
15	Frequent geological hazards	5, 9, 14	8, 9
16	Narrow construction site	3, 15	1–10
17	Harsh climatic conditions	4, 7	4, 7, 8, 9, 10
18	Lack of social and peripheral acceptance	13, 15	9, 10
19	Inadequate price realization mechanism for TI output	16	2, 3, 5
20	Excessive TI targets	1, 13, 15	9, 10
21	Insufficient stock of information related to TI	15	1, 2, 3, 4
22	Disconnect between TI and project reality	7, 9	6, 7
23	Difficulty in transporting materials	5, 8	1, 4–10
24	Shortage of management, technology, and talent	13, 14	1, 2
25	Low level of resource input	8, 9, 10	5, 6
26	Inadequate use of knowledge resources	2, 11, 12	1–10
27	Temporary and dispersed TI organizations	15	1–10
28	Large project size	5, 15	1–10
29	High level of risk management	11, 16	1–10

**Table 4:** The coding process of RB-TI in CMDAs.

No.	Intermediate coding	Initial coding
1	Demands of survey and design TI	Wind-resistant design
2	Demands of survey and design TI	Seismic design
3	Demands of survey and design TI	Environmental design
4	Demands of survey and design TI	Anti-fatigue design
5	Demands of construction TI	Main cable erection
6	Demands of construction TI	Strong wind construction
7	Demands of construction TI	Optimization of materials and equipment
8	Demands of construction TI	Deep water construction
9	Demands of construction TI	Eco-friendly construction
10	Demands of construction TI	Anchor construction
11	Demands of construction TI	Monitoring and measuring
12	Demands of maintenance TI	Corrosion protection
13	Demands of maintenance TI	Integration of construction and maintenance
14	Demands of maintenance TI	Emergency plans
15	External environmental obstacles	Frequent geological hazards
16	External environmental obstacles	Narrow construction site
17	External environmental obstacles	Harsh climatic conditions
18	External environmental obstacles	Lack of social and peripheral acceptance
19	External environmental obstacles	Inadequate price realization mechanism for TI output
20	Technology management obstacles	Excessive TI targets
21	Technology management obstacles	Insufficient stock of information related to TI
22	Technology management obstacles	Disconnect between TI and project reality
23	Resource use obstacles	Difficulty in transporting materials
24	Resource use obstacles	Shortage of management, technology and talent
25	Resource use obstacles	Low level of resource input
26	Resource use obstacles	Inadequate use of knowledge resources
27	Organization management obstacles	Temporary and dispersed TI organizations
28	Organization management obstacles	Large project size
29	Organization management obstacles	High level of risk management

**Table 5:** TI demands and obstacles of the LD Bridge and corresponding module design.

TI demands and obstacles	Specific analysis	Module design
Wind-resistant design	High average wind speed and large wind angle of attack	TI module of canyon wind resistance
Seismic design	Large seismic intensity near the fault	TI module of strong seismic resistance in the near field area
Environmental design	Located in a highland ecological reserve	TI module of environmental protection
Deep water construction	The Dadu river is over 10 meters deep and fast-flowing	TI module of deep water operation
Anchor construction	The main cable force of a single anchor of tunnel anchor is up to 4.6 tons	TI module of the construction of large tunnel anchors
Narrow construction site	Both banks of the mountain are exposed rock and steep	TI module of steep slope construction
	The site in the gorge is too narrow to lift stiffening beams from the valley floor	TI module of stiffened beam section lifting
Integration of construction and maintenance	Harsh environment and difficult post-operation and maintenance	TI module of structural durability
Difficulty in transporting materials	Weak infrastructure, large variety, and volume of material requirements	Modular management measures
Large project size	Thousand-meter railway suspension bridge with a large span	
High level of risk management	Geological risk, construction safety risk, duration risk, environmental risk, and social risk	

## Data Availability

All datasets generated for this study are included in this paper.
